The article "Distribution and Risk Factors of Multidrug-Resistant Bacteria Infection in Orthopedic Patients" was published in 2022. Journal: J Healthc Eng.

# Distribution and Risk Factors of Multidrug-Resistant Bacteria Infection in Orthopedic Patients

**DOI:** 10.1155/2022/2114661

**Published:** 2022-01-27

**Authors:** Maohua Liang, Qiang Liu

**Affiliations:** ^1^Orthopcdics Department of Tai'an Central Hospital, Tai'an, Shandong 271000, China; ^2^The University of Georgia, Athens, GA, USA

## Abstract

**Objective:**

To study the distribution and risk factors of multidrug-resistant bacteria (MDROS) infection in orthopedic patients and to provide reference for clinical prevention and control measures.

**Methods:**

The data of 239 inpatients with orthopedic trauma from June 2019 to December 2020 were selected as the research objects, and the distribution characteristics of MDROS infection were analyzed through the real-time monitoring system of nosocomial infection. Logistic regression analysis was used to screen out the risk factors causing MDROS infection, and the preventive measures were put forward.

**Results:**

178 strains of pathogens were isolated from 239 patients, including 53 strains of MDROS, and the detection rate was 29.78%. The main pathogenic bacteria were ESBLs, MRSA, CRAB, CRE, and MDR/PDRPA. The main infection sites of MDROS in orthopedic patients were the respiratory tract and wound. No CRE1 was detected, and 64.39%, 17.42%, and 14.39% of ESBL-producing bacteria, MRSA, and MDR/PDRPA, respectively, were detected. Logistic multivariate analysis showed that the length of hospital stay, antibiotic use time, open injury, and serum albumin level were independent risk factors of MDROS infection in orthopedic trauma patients.

**Conclusion:**

To prevent MDROS infection in orthopedic patients, we should start from many aspects, focusing on reducing unnecessary hospitalization days, rationally preventing the use of antibacterial drugs, effectively treating basic diseases, etc., timely and effective thorough debridement, strengthening functional training, reducing bed rest, and strengthening targeted monitoring of related infections which are the keys to reduce MDROS infection in orthopedic patients.

## 1. Introduction

Multidrug-resistant bacteria refer to pathogenic bacteria with multidrug resistance, and it has drug resistance to a variety of drugs. They are defined as microorganisms against three categories (such as aminoglycosides, macrolides, and *β*-lactams) or more than three kinds of antibiotics with different mechanisms which are resistant at the same time, rather than three kinds of the same kind. P-resistance is a pan-resistant strain, which is resistant to almost all kinds of antibiotics, such as pan-resistant *Acinetobacter*, aminoglycosides, penicillins, cephalosporins, carbapenems, tetracyclines, fluoroquinolones, and sulfonamides.

Multidrug-resistant bacteria (MDROS) are a kind of pathogenic bacteria which are resistant to three or more antibiotics at the same time. In recent years, with the increasing drug resistance of pathogenic bacteria, MDROS has gradually become an important pathogen of open wound infection in orthopedics, which increases the difficulty of using antibiotics to treat open wound infection in orthopedics, and has become a thorny clinical problem [1, 2]. Monitoring and analyzing the distribution characteristics and risk factors of MDROS in orthopedic patients can provide reference for the prevention and treatment of MDROS infection in orthopedic patients [3]. In order to effectively reduce the incidence of MDROS in open wounds in orthopedics, this study reviewed the risk factors of MDROS infection in open wounds in orthopedics and provided reference for preventing MDROS infection in open wounds in orthopedics.

## 2. Literature Review on the Etiology of Orthopedic Infection

Bacterial drug resistance refers to the relative resistance of bacteria to certain antibacterial drugs (antibiotics or disinfectants). The drug resistance of bacteria is the result of evolutionary selection of bacteria, and the abuse of antibiotics aggravates the generation of drug resistance of bacteria. Because antibiotics can effectively eliminate or slow down the growth of bacteria, they play an important role in preventing and controlling infectious diseases. Therefore, in the current treatment of bacterial infection, doctors and patients are overreliant on them. After obtaining drug resistance, the treatment is difficult, the effective rate of treating infected people is reduced, the mortality rate is increased, and the medical expenses will rise sharply. Therefore, understanding the progress of bacterial variation, drug resistance system and treatment play a key role in guiding the clinical application of antibacterial drugs.

The most common bone injury is fracture, which refers to the interruption of continuity or integrity of the bone or trabecula. According to the connectivity between the fracture and external environment, we can divide traumatic fracture into two types: closed and open. After a long period of evolution, the coding structural protein of drug-resistant strains changed due to chromosome deletion and breakage, and DNA fragments containing drug-resistant genes spread drug resistance among strains after being transferred and inserted into the drug-resistant plasmid. According to the test data of Birson et al. [4], among all the isolated bacteria, Gram-negative bacilli accounted for the majority, accounting for 59.9%. Among them, they are mainly divided into *Pseudomonas aeruginosa* and *Acinetobacter*. According to the research data of Li et al. [5], the use frequency of certain antibiotics by clinicians may affect the drug resistance of bacteria. The higher the frequency of use, the higher the resistance of bacteria to these drugs, such as the third-generation cephalosporins. The lower the frequency of use, the lower the resistance of bacteria to such drugs, such as ciprofloxacin.

Integrons are contained in bacteria, which can recognize and capture mobile gene boxes. In addition, there are also site-specific recombinant expression systems, especially Gram-negative bacteria genes. Antibiotics must be injected at one time in a whole day's dose. This is not only conducive to better display of curative effect but also can effectively reduce toxic and side effects. According to the research data of Yang and others [6], as far as *Staphylococcus aureus* is concerned, it is not only very resistant to penicillin but also to erythromycin, gentamicin, and sulfamethoxazole. In the coagulase test, some staphylococci were negative. In the examination of surgical specimens, the results show that compared with aerobic bacteria, the detection rate of anaerobic bacteria is higher, probably in the range of 55%–75% [7]. It was found that, in the last 20 years, the local concentration of antibiotics was generally higher, but the serum concentration was lower, so they became an effective choice for treating infection in orthopedic surgery [8].

## 3. Materials and Methods

### 3.1. General Information

The clinical data of patients with the same strain who were diagnosed positive twice were used in the diagnosis of infection. The patients were divided into the MDRB group and non-MDRB group. The basic conditions of the two groups were recorded and analyzed, such as basic diseases, invasive operation, drug sensitivity of MDRB beads, mechanical ventilation (noninvasive), smoking, admission to the intensive care unit, and long-term bed rest. From June 2019 to December 2020, 239 patients with open wound infection were treated, including 89 patients with MDRO infection, 51 males and 38 females, with an average age of 49.32 ± 19.53 years from 4 to 81 years old, and 150 patients with non-MDRO infection, 109 males and 41 females, with an average age of 55.37 ± 15.03 years from 3 to 85 years old.

### 3.2. Inclusion and Exclusion Criteria

The inclusive criteria were as follows: methicillin-resistant *Staphylococcus aureus* (MRSA), vancomycin-resistant *Enterococcus* (VRE), extended spectrum lactamase (ESBL) producing *Escherichia coli* and *Klebsiella pneumoniae*, carbapenem-resistant Enterobacteriaceae (CRE), carbapenem-resistant *Acinetobacter baumannii* (CRAB), multidrug-resistant/pan drug-resistant *Pseudomonas aeruginosa* (MDR) isolated and identified from orthopedic clinical infection samples/PDRPA, and other common MDROs.

The exclusion criteria were as follows: exclusion of MDROs colonized uninfected, noninfectious inflammation, and MDRO-contaminated samples.

### 3.3. Method

Sputum samples of patients were collected and identified by using the VITEK-2 automatic bacterial identification instrument. Drug sensitivity test was carried out by the K-B method, and the results were judged according to the CLSI standard [9].

The infection management department full-time personnel were responsible for monitoring with the help of the relevant departments of the hospital. Factors that might be related to MDROS infection were registered and analyzed in detail: gender, age, hospitalization time, ventilator use time, indwelling catheter time, central venous intubation time, presence of underlying diseases, types of antibacterial drugs used, immunosuppressive agents used, and operation history.

### 3.4. Statistical Analysis

Excel 2013 tables were used to sort out the data, and SPSS 19.0 software was used for univariate and multivariate logistic regression analyses of the data. *P* < 0.05 indicated a statistically significant difference.

## 4. Results

### 4.1. Univariate Analysis of Risk Factors for MDROS Infection

178 strains of pathogens were isolated from 239 patients, including 53 strains of MDROS, and the detection rate was 29.78%. The main pathogenic bacteria were ESBLs, MRSA, CRAB, CRE, and MDR/PDRPA. The main risk factors were the patient's age, hospital stay, operation time, antibiotic use time and glucocorticoid use, complicated diabetes, open injury, mechanical ventilation, serum albumin, and indwelling catheterization. The differences were statistically significant within the same group (*P* < 0.05).

### 4.2. Distribution of MDROS-Infected Sites

The respiratory tract and wound were the main sites of MDROS infection in orthopedic patients. No VRE was detected, and the percentages of ESBLS-producing bacteria (ESBLS being the CRE1 strain at the same time), MRSA, and MDR/PDRPA were 64.39%, 17.42%, and 14.39%, respectively, as shown in Table 1.

### 4.3. Logistic Multivariate Analysis of MDROS Infection

Logistic multivariate analysis showed that the length of hospital stay, antibiotic use, open injury, and serum albumin were all independent risk factors for MDROS infection in orthopedic trauma patients. The results of the logistic multivariate analysis of MDROS infection are shown in Table 2.

## 5. Discussion

MDROS infection has become a global public health problem and clinical challenge. The prevention and control of MDROS is currently one of the biggest challenges in infection control. In recent years, the infection of MDROS in different countries and regions has been increasing [10, 11]. Through *χ*^2^ test statistics, it was found that, except for age and combined cardiovascular disease and MDROS infection in orthopedic trauma patients, there was no significant correlation, and the other factors were significantly correlated with MDROS infection in orthopedic trauma patients (*P* < 0.05). In this study, 178 pathogens were isolated from 239 orthopedic patients, including 53 MDROS strains, with the detection rate of 29.78%. The respiratory tract and wound were the main sites of MDROS infection. The percentages of ESBLs, MRSA, and MDR/PDRPA were 64.39%, 17.42%, and 14.39%, respectively, indicating that the infection of MDROS in open wounds of the orthopedics department was increasing, especially in the respiratory tract, wound, and incision.

In this study, univariate regression analysis was performed on 17 possible risk factors for MDROS infection in open orthopedic wounds, including age, gender, hospital stay, use of glucocorticoids, concomitant underlying diseases and comorbidities, wound types, prevention and use of antibacterial drugs, the time and number of antibacterial drugs used, and whether or not they were used. The results showed that three factors, except age, gender, and prevention and use of antibacterial drugs before debridement, were not related to MDROS infection in open orthopedic wounds (*P* > 0.05), suggesting that rational prevention and use of antibacterial drugs before debridement could reduce MDROS infection in open orthopedic wounds. Patients with diabetes, chronic obstructive pulmonary disease, and open injury in orthopedics have a higher infection rate of MDROS than patients without the above diseases, and these patients have low immune function and impaired defense function and are prone to infection with MDROS. Multivariate unconditional logistic regression analysis showed that hospitalization time, ventilator use time, central venous intubation time, and basic disease were the independent risk factors for MDROS infection, which increased the risk of MDROS infection by 1.022 times, 2.149 times, 1.347 times, and 0.639 times, respectively.

This pilot study also showed that the frequency of hospitalizations for the same wound infection was also a risk factor for MDROS infection in orthopedic patients. It is easy to cause exogenous infection when carrying out patient care or contacting patients. Exogenous infection is mostly caused by external factors such as medical care. It is generally believed that the transmission of pathogens between patients (including direct transmission and transmission mediated by medical devices and medical staff) and the improper use of antibiotics are the two major risk factors of exogenous nosocomial infection. Whether there are perfect handwashing and disinfection facilities in the hospital, whether medical waste is strictly distinguished, whether medical care follows strict operation specifications, and whether all invasive treatments and care ensure sterility may cause nosocomial infection. Therefore, it is difficult for hospitals to control the occurrence conditions of endogenous infection, and exogenous infection has become the focus of prevention and control. ICU patients are in a more severe condition, and the longer they stay in the hospital, the more likely they will be exposed to MDROS [12]. Traumatic diagnosis and treatment can damage the body defense barrier and increase the chance of MDROS infection in patients. Long-term use of glucocorticoids, hemoglobin, and decreased serum albumin concentration can reduce its immune function, and it is also one of the important causes of MDROS infection in orthopedics. Long-term use of glucocorticoids, increased blood glucose, and decreased hemoglobin and plasma albumin can reduce the immune function of patients and also serve as an important incentive for MDROS infection [13, 14]. The main cause of stroke-related pneumonia triggered by consciousness disorder is aspiration, which leads to a large amount of oropharyngeal secretions' aspiration into the human lung and induces the breeding of drug-resistant bacteria. At the same time, patients with the disorder of consciousness need to undergo invasive operations such as sputum aspiration and indwelling catheter to allow external pathogens to enter the patient's body, causing pulmonary infection.

Therefore, the prevention of MDROS infection in orthopedic patients should be started from multiple aspects, with the focus on reducing unnecessary hospital stays, rational prevention and use of antibacterial drugs, effective treatment of underlying diseases, timely and effective thorough debridement, strengthening functional exercise, and reducing bed rest as the key [15]. In accordance with the principle of aseptic manipulation, isolation signs should be hung at the gate of the ward, the bedside card, and the patient information list as required to remind the patients of the MDROS infection. In addition, the rehabilitation process should be strengthened, which will also lead to a significant increase in medical expenses and excessive occupation of health service resources.

## 6. Conclusion

In summary, pathogen detection and drug sensitivity test in the treatment of orthopedic patients can improve the pertinence and effectiveness of the treatment and avoid blind medication. We should strengthen the hardware construction of operating rooms in primary hospitals, improve the professional quality of medical staff, strictly standardize the operation procedures, improve the sense of responsibility of relevant personnel, and enhance the patients' awareness of sterility and nutritional status of the body in order to effectively reduce the occurrence of postoperative infection and complications. MDROS infection is relatively easy to occur in orthopedic trauma patients, and active prevention and control measures should be taken to effectively avoid the occurrence of MDROS infection.

## Figures and Tables

**Table 1:** Distribution of MDROS-infected sites and detection constituent ratio in orthopedic patients (%).

MDROS	Infected site						Total	
	Wound	Surface of a wound	Incision	Urinary tract	Respiratory tract	Others	Number of patients	Constituent ratio
ESBLs	4	11	14	8	46	2	85	64.39
MRSA	8	13	1	0	0	1	23	17.42
MDR/PDRPA	4	10	0	0	4	1	19	14.39
CRAB	0	0	1	1	3	0	5	3.79
Total	16	34	16	9	53	4	132	100

**Table 2:** Logistic multivariate analysis of MDROS infection.

Risk factor	*β* Value	*SE* Value	Ward *x*^2^	*P* Value	*OR* Value	95% CI
Inpatient days	0.207	0.117	4.241	<0.05	1.172	1.027–3.395
Open injuries	1.371	1.239	6.572	<0.05	3.662	1.375–9.621
Antibiotic usage time	0.556	0.826	5.330	<0.05	1.605	1.457–4.523
Serum albumin level	1.261	0.772	6.821	<0.05	1.961	1.093–3.012

## Data Availability

The data used to support the findings of this study are included within the article.
